The article "Clinical Study on the Evaluation of the Condition of Patients with Gastric Tumors and the Choice of Surgical Treatment by Gastric Ultrasonic Filling Method" was published in 2022. Journal: Contrast Media Mol Imaging.

# Clinical Study on the Evaluation of the Condition of Patients with Gastric Tumors and the Choice of Surgical Treatment by Gastric Ultrasonic Filling Method

**DOI:** 10.1155/2022/3960929

**Published:** 2022-06-09

**Authors:** Sainan Wang, Yun Hong, Lizong Wang

**Affiliations:** ^1^Ultrasonic Medical Department, The First Affiliated Hospital of Wannan Medical College, Wuhu, Anhui 241000, China; ^2^General Practice Department, The First Affiliated Hospital of Wannan Medical College, Wuhu, Anhui 241000, China

## Abstract

Objective. To explore the clinical value of the gastric ultrasonic filling method in evaluating the condition of patients with gastric tumors and guiding the selection of treatment methods, provide data support for clinical gastric filling ultrasonography in the evaluation of gastric cancer patients, and provide the basis for the choice of surgical treatment. *Methods*. This study retrospectively analyzed 50 patients with gastric cancer treated in our hospital from April 2017 to January 2022. All 50 patients were examined by the gastric ultrasound filling method. The TNM staging results of gastric cancer were analyzed with the results of gastroscopic biopsy or postoperative pathological examination as the diagnostic gold standard. *Results*. The ultrasonic detection rate of 50 patients with gastric cancer was 94.00% (47/50). Among them, 3 cases missed diagnosis were of early intramucosal carcinoma, which were only diagnosed as erosive gastritis. 1 case was located in the gastric body, and the other 2 cases were located in the gastric antrum. Ultrasound assessment of gastric mucosal thickness in T1-T2 stage was 9.8 mm, which was significantly lower than that in T3-T4 stage, which was 17.0 mm (*p* < 0.05). The diagnostic accuracy of the gastric ultrasound filling method in the diagnosis of T1, T2, T3, and T4 was 41.67%, 57.14%, 96.00%, and 83.33%, respectively. The total diagnostic accuracy of T-stage was 76.00% (38/50). The total judgment rate of too shallow and too deep was 10.00% and 14.00%, respectively. The diagnostic accuracy of the gastric ultrasound filling method was 88.89%, 81.81%, 70.00%, and 82.00%, respectively. The diagnostic accuracy of the gastric ultrasound filling method in the diagnosis of M0 and M1 stages was 100.00%, and the total diagnostic accuracy of the M-stage was 100.00%. The ROC curve drawn by GFUS in the diagnosis of T-stage of gastric cancer had three components: the specificity was the horizontal axis, the sensitivity was the vertical axis, and the area under the curve was 0.978. The difference was statistically significant (*p* < 0.05). *Conclusion*. Before the operation of patients with gastric cancer, using the gastric ultrasonic filling method and ultrasonic examination method to diagnose them can timely clarify the clinical stage of patients, so that clinicians can choose the most appropriate operation method according to their clinical stage, which is worthy of popularization and application in clinic.

## 1. Introduction

Cancer is a major public health problem worldwide, according to the latest cancer statistics from the American Cancer Society (ASC) in 2021 estimated 1.9 million new cancer cases and 610,000 cancer deaths in the United States [1]. According to the 2018 GLOBOCAN report data, there are about 18.1 million new cancer patients and 9.6 million deaths from cancer in the world every year. Among them, the annual increase in gastric cancer is 1.033 million, ranking fifth in the global incidence of malignant tumors [2, 3]. In 2020, 769,000 people died of gastric cancer in the world, and the new gastric cancer cases and deaths in China accounted for 43.9% and 48.6%, respectively [4]. According to the registration data of malignant tumors in 2015, there were about 403,000 new cases of gastric cancer in my country. The incidence rate ranks second among malignant tumors, and with 291,000 deaths, the mortality rate ranks third among malignant tumors in China [5, 6]. Because the clinical manifestations of early gastric cancer are not obvious or even without any symptoms, patients are easy to ignore. Most patients have developed advanced gastric cancer when they are diagnosed in the hospital, and the clinical cases have also developed to stage III or IV accounting for more than half [2]. Most of the clinical treatment is based on the clinical stage of the patient, and the most suitable surgical method is selected for the treatment. Therefore, only by diagnosing the clinical stage of such patients before surgical treatment can we ensure the therapeutic effect of surgery and improve the quality of life of patients.

In recent years, with the rapid development of computer technology, the continuous enhancement of ultrasound technology, and the emergence of various digital processing and ultrasound probes, ultrasound technology has been widely used in the medical field and has achieved gratifying results. Until today, ultrasound examination has become a clinical. It is one of the indispensable means of diagnosing certain diseases [7]. However, in the digestive tract organs such as the gastrointestinal tract, the use of ultrasound has encountered great limitations and doubts. Using it will cause considerable interference, so it will greatly hinder the display of images formed by ultrasonic waves, especially in terms of clarity. It is precisely because of the above reasons that before the 1980s, it was agreed at home and abroad that the ultrasound examination of the gastrointestinal tract was basically a blind spot [8], which did not receive due attention and development. It was not until the introduction of gastrointestinal ultrasound contrast agents, which greatly improved the imaging performance of gastrointestinal ultrasound, that gastrointestinal ultrasound was rapidly applied and developed, and gradually became an important means of diagnosing gastrointestinal diseases, Wang et al. [9] pointed out that gastric filling ultrasonography has a high diagnostic value in gastroesophageal reflux disease. Currently, gastric filling ultrasonography (GFUS) has been widely used in the preoperative evaluation of gastric cancer. It can not only understand the location and size of the lesion but also preliminarily judge the nature of the lesion, and can also observe the scope and degree of infiltration of the lesion and surrounding organs [10, 11]. But there are few reports on the application of GFUS to the clinical staging of gastric cancer patients before surgery, and there are few reports on the evaluation of the patient's condition. The ultrasonography results and TNM staging of gastric cancer patients were analyzed and compared with postoperative pathological results in order to explore the clinical application value of gastric filling ultrasonography in the evaluation of gastric cancer patients and the selection of surgical treatment methods.

## 2. Materials and Methods

### 2.1. General Information

A retrospective analysis was conducted of 50 patients who were diagnosed with gastric cancer in our hospital from April 2017 to January 2022. Inclusion criteria: (1) patients with gastric cancer; (2) patients with preoperative GFUS and complete staging data; (3) patients undergoing surgery. Exclusion criteria: (1) patients with missing pathological data; (2) patients with gastric stromal tumor; (3) patients suffering from severe mental illness and cognitive impairment; (4) patients with dysfunction of liver and kidney function; and (5) patients with coagulation dysfunction. There were 22 males and 28 females; the average age was 25.5 ± 25 years old; tumor location: upper stomach in 20 cases, middle stomach in 11 cases, and lower stomach in 19 cases. There were 12 cases of early gastric cancer and 38 cases of advanced gastric cancer. Among the 50 patients with gastric cancer, 48 underwent subtotal gastrectomy or endoscopic mucosal resection, and 2 underwent palliative surgery. The study has been approved by the hospital's ethics committee, and all patients have informed consent.

### 2.2. Ultrasonic Examination

All 50 patients were examined with MINDRAY Resona 7T. The frequency of the convex array probe was 3.5∼5.0 Hz and the frequency of the high-frequency linear array probe was 7.5∼12 Hz. Before the examination, ask the examinee not to eat or drink water for 8 h, guide them to take oral display aids to fill the gastric cavity for examination, and guide the patients to take different body positions for examination, such as supine position, left-lying position, right-lying position, and semisitting position. According to the projection of gastroduodenal body surface, ensure that the sonograms of gastric cardia, gastric bottom, gastric body, gastric antrum, duodenal bulb, and horizontal part are clearly presented, and scan the surrounding tissues to observe whether there is lesion metastasis. Record the location, scope, and depth of the lesion. Gastric ultrasound enhancer (Huzhou East Asia Pharmaceutical Products Co., Ltd.): sound velocity is 1545 m/s and acoustic impedance rate is 1.58 × 10.5 Pa.s/m, sound attenuation coefficient is 1.68 db/(cm. MHz), and viscosity is 123 MPa s. The pH value is 6.24. Make it into a paste solution in strict accordance with the production instructions. When the patient's stomach is full, the ultrasonic image will show five layers of gastric wall structure. The first layer is the strong echo line (gastric mucosal surface layer), the second layer is the low echo line (mucosal lamina propria-mucosal muscle layer), the third layer is the strong echo line (gastric mucosal muscle layer-submucosa), the fourth layer is the low echo line (intrinsic muscle layer), and the fifth layer is the strong echo line (plasma mucosal layer and surrounding tissues).

### 2.3. Gastroscopy

Gastroscopy uses the olympus CV 290 (host model: GIFH290) to observe the duodenal bulb from the pharynx in turn. After finding the lesion, determine the location, size, and scope and then observe the boundary, glandular duct, and microvessel of the lesion by the electronic staining method, and conduct an accurate biopsy under its guidance.

### 2.4. Ultrasonic Classification Standard of Gastric Cancer

The diagnostic classification is based on Borrmann's gross morphological classification: the type of mass is that the mass bulges into the stomach and it is concave convex. The limited ulcer type has a large ulcer area, the edge is in the shape of a river bank, and the boundary between the lesion and the normal gastric wall is obvious. The infiltrating ulcer type is the ulcer in which the adjacent gastric wall thickening area is large, and the whole is in the shape of crater. The diffuse infiltrative type is characterized by the expansion of the scope of pathological changes entering the gastric wall and the complete disappearance of the layers. The TNM staging criteria for gastric cancer is as follows: Tis: carcinoma in situ; T1: tumor infiltrates basement membrane or submucosa; T2: tumor infiltrates the muscular layer or subserosal layer; T3: the tumor penetrates the serosa (visceral peritoneum) but has not infiltrated the adjacent organs; T4: tumor infiltrates adjacent organs; N0: no local lymph node metastasis; N1: 1∼6 local lymph node metastases; N2: 7∼15 local lymph node metastases; N3: more than 15 local lymph node metastases; M0: no distant metastasis; and M1: distant metastasis.

### 2.5. Statistical Methods

SPSS 26.0 statistical software is used for data analysis. The measurement data are expressed in median (range), the rank sum test was used to compare the two groups, and the counting data are expressed in (*n*, %). The ROC curve was drawn by GFUS to diagnose the T-stage of gastric cancer, and the area under the curve (AUC) was obtained to evaluate the diagnostic efficiency of GFUS in diagnosing the T-stage of gastric cancer.

## 3. Results

### 3.1. Ultrasonic Diagnosis and Pathological Results of Gastric Cancer

The ultrasonic detection rate of 50 patients with gastric cancer was 94.00% (47/50). Among them, 3 cases missed diagnosis of early intramucosal carcinoma, which were only diagnosed as erosive gastritis. One case was located in the gastric body, and the other 2 cases were located in the gastric antrum (see Table 1).

### 3.2. Ultrasonic T-Stage Diagnosis Results

The diagnostic accuracy of T1, T2, T3, and T4 was 41.67%, 57.14%, 96.00%, and 83.33%, respectively. The total accuracy of T-stage diagnosis was 76.00% (38/50), the total shallow judgment rate was 10.00%, and the total deep judgment rate was 14.00% (see Table 2). The ROC curve was drawn by GFUS for the diagnosis of gastric cancer at T-stage. The specificity was on the horizontal axis and the sensitivity was on the vertical axis. The area under the curve was 0.978, and the difference was statistically significant (*p* < 0.05). As shown in Figure 1 the ultrasound assessment of gastric mucosal thickness in T1-T2 stage was 9.8 mm, which was significantly lower than that in T3-T4 stage, which was 17.0 mm, and the difference was statistically significant (*p* < 0.05) (see Table 3).

### 3.3. Accuracy of Ultrasonic N-Stage Diagnosis

The diagnostic coincidence rates of N0, N1, N2, and total were 88.89%, 81.81%, 70.00%, and 82.00%, respectively. No stage N3 lymph nodes were found (see Table 4).

### 3.4. Accuracy of Ultrasonic M-Stage Diagnosis

Ultrasonography showed liver metastasis in 3 cases and peritoneal metastasis in 3 cases. The coincidence rate of M0 and M1 ultrasonography was 100% (see Table 5)

### 3.5. Selection of Surgical Treatment

The main operative methods selected in this group were endoscopic submucosal dissection, standard radical resection, and extended radical resection. The treatment of TLA is mainly endoscopic submucosal dissection, while the treatment of TLB is mainly radical surgery. The resection of lesions is divided into whole resection, complete resection, radical resection, and curative resection. There are atypical cells on the edge, and basal or partial resection is performed. Standard radical gastrectomy for gastric cancer is to remove 2/3 of the proximal and distal stomach or the whole stomach according to the size and location of the tumor, plus N2 lymph node dissection, that is, D2 radical gastrectomy. Extended radical resection refers to the fact that primary or metastatic cancer directly invades the perigastric organs and the invaded organs must be jointly removed before radical resection, or lymph node metastasis above N2 is positive, and lymph node dissection above D2 or D3 must be performed before grade B radical resection can be obtained. According to the stage determination results, radical operation of D2 or D2 + 12 group lymph node dissection was selected for IB, II, IIIa, and some IIIB cases. Extended radical resection was selected for some stage IIIB and IV cases. If stage IV patients have no radical significance, simple gastrojejunostomy and exploratory laparotomy are routinely performed.

## 4. Discussion

The incidence rate of China's gastric cancer is 42.6% (12). According to the latest statistics of the China National Cancer Center in February 2018, although the overall incidence rate of gastric cancer is decreasing, gastric cancer is still the second place malignant tumor in China, second only to lung cancer (3). The pathogenesis of gastric cancer is complex, which is mainly related to environmental, genetic, immune, infection, and other factors. Most of the patients are people with bad eating habits, a family history of gastric cancer or *Helicobacter pylori* infection [12–14]. According to the progress of the disease, it can be divided into early gastric cancer and middle and late gastric cancer. The former lesions are mostly in the mucosa or submucosa. The types of lesions can be divided into protuberant, shallow phenotype, and concave type, without typical clinical symptoms. The lesions of the latter have invaded the muscle layer or the whole layer and even metastasized in severe cases. The types of lesions can be divided into ulcer type, mushroom umbrella type or polypoid type, invasive type, and mixed type. The clinical symptoms are mainly abdominal tenderness, jaundice, and distant lymph node metastasis [15, 16]. The treatment methods of the disease mainly include surgery, radiotherapy, and chemical drug treatment. The surgical treatment mainly selects radical surgery or nonradical surgery according to the patient's own situation [17].

TNM staging is one of the staging forms of tumors, in which T represents the primary focus, *n* represents lymph nodes, and M represents distant metastasis. The later the TNM staging is, the more serious the condition is, the more complex and difficult the treatment is, and its treatment effect will also be affected [18]. Therefore, the clinical diagnosis of the disease severity of gastric cancer patients can be based on the TNM stage, which is helpful in providing a good reference for the follow-up surgical treatment. The usual clinical diagnosis of TNM stage of gastric cancer mostly adopts abdominal ultrasound, CT, and MRI to examine patients. This kind of examination method has high sensitivity to the M-stage but low sensitivity to the T and N stages. It is unable to determine the depth of invasion of gastric cancer in the digestive tract wall, and the judgment effect of metastatic lymph nodes is poor, and the overall effect is not good. The early occurrence and treatment of gastric diseases can greatly improve the prognosis of patients. Gastroscopy is considered to be the first choice for the diagnosis of gastric diseases. However, as an invasive examination, gastroscopy has many problems, such as discomfort, mucosal injury, aspiration, and so on. Relatively speaking, ultrasonography is a convenient, noninvasive, and economical examination method, but due to the interference of gas in the gastrointestinal tract, its application in the diagnosis of gastrointestinal diseases is often limited [19]. Warren et al. [20] first used hydrophilic methylfibronectin oral suspension to fill the stomach in ultrasonography in 1978. Retroperitoneal organs such as the pancreas underwent ultrasonography. Since then, researchers have conducted many studies on oral gastrointestinal adjuvants [21, 22]. The echogenic gastrointestinal ultrasound aid used in this study takes coix seed as the main component and presents a uniform medium echo in the filled stomach. It can clearly show the normal level and lesion area of the gastric wall, determine the origin, morphology, infiltration degree, scope of the lesion, and other relevant morphological information, and observe the peristalsis of the gastric wall. And it has the advantages of slow emptying and is easy to be accepted by children and the elderly.

### 4.1. Diagnosis of Gastric Cancer by Gastric Filling Ultrasonography

Ultrasonic examination of the stomach has been delayed, and the image of the stomach has been delayed. In recent years, with the improvement of gastric window ultrasound AIDS, the images of gastric cancer have been significantly improved. The diagnostic value of ultrasonography in gastric cancer has been gradually recognized. In this study, after the gastric cavity was evenly filled with a paste echo gastric contrast agent, the uniform echo area formed by the contrast agent in the cavity formed an obvious contrast with the gastric wall and surrounding tissues. Taking this as the sound transmission window, we can clearly observe the five-layer structure of the gastric wall and judge the depth of tumor infiltration into the gastric wall, the invasion of surrounding organs, and lymph node metastasis. Gastric cancer is characterized by decreased and thickened echo of gastric wall, unclear display of five-layer structure of gastric wall, interruption of continuity of mucosal layer, formation of ulcer or mass, etc (see Figure 1). This study found that the results of ultrasonic examination and pathological examination of gastric filling for gastric ulcer and gastric malignant tumor were accurate. The ultrasonic detection rate of 50 patients with gastric cancer was 94.00% (47/50), which was basically consistent with the results of many studies using the chi square test to compare gastric filling ultrasonic examination and gastroscopy [23–25]. However, it should be noted that 3 cases missed in the report of gastric filling ultrasonography were early intramucosal carcinoma, which were only diagnosed as erosive gastritis. One case was located in the gastric body, and the other 2 cases were located in the gastric antrum. Moreover, it is of the shallow depression type. The reason may be that after the stomach is fully filled, the gastric mucosa is excessively flattened, which makes it difficult to display small ulcers, resulting in the diagnosis of erosive gastritis. At this time, the operator's experience and skills are very important.

### 4.2. T-Stage Diagnosis of Gastric Cancer by Gastric Filling Ultrasonography

It can be seen from Table 2 that the diagnostic coincidence rates of T3, T4 and total are high, and the diagnostic coincidence rate of T1 is the lowest. The ROC curve drawn by GFUS in the diagnosis of T-stage of gastric cancer had three components: the specificity was the horizontal axis, the sensitivity was the vertical axis, and the area under the curve was 0.978. The difference was statistically significant (*p* < 0.05). In this group, the judgment rate of too shallow was 10.00%, and 3 cases of T1 gastric cancer were not detected. The cause of too shallow judgment may be related to the location of the lesion. After filling the gastric cavity with the developer, the satisfaction rate of far-field display can reach 97%, and the dissatisfaction rate of near-field display is 30%. The developer can not eliminate the near-field artifacts. When using the most commonly used oblique coronal scan, the greater curvature of the stomach is just located in the near-field. In addition, the skill and proficiency of the operator are also very important. When finding a lesion and judging its infiltration depth, it is necessary to conduct continuous scanning in multiple sections, including coronal oblique section, long axis section, and short axis section, because the postoperative pathological tissue section is a pathological diagnosis made after continuous multipoint sampling, and the stages of different parts of a cancer may be different, However, the operator must make the final T-stage according to the position with the maximum infiltration depth to avoid too shallow judgment. The judgment rate of over depth in this group was 14.00%. Among 12 cases of T1 gastric cancer, 4 cases of over depth were judged as T2, and 2 cases of 3 cases of T2 gastric cancer were judged as T3. The over depth judgment occurred in T1 and T2. The causes of T1 stage excessive depth may be the inflammatory reaction around the focus, the fibrosis of adjacent tissues, and the surrounding scar tissue, showing the weakly echoic mass with thickened gastric wall in the sonogram, which makes the real tumor boundary difficult to distinguish. The judgment of excessive depth in the T2 phase may also be related to the loss of serosa in some parts of the gastric wall [26]. In addition, the results of this study pointed out that the median gastric mucosal thickness in T_1_-T_2_ stages assessed by ultrasound was 9.8 mm, which was significantly lower than the median gastric mucosal thickness in T_3_-T_4_ stages, which was 17.0 mm (*p* < 0.05). It is suggested that gastric mucosal thickness may be used as an indicator for gastric filling ultrasonography to judge gastric cancer staging, and the results are similar to those of Liu et al. [25].

### 4.3. N-Stage Diagnosis of Gastric Cancer by Gastric Filling Ultrasonography

The results of gastric filling ultrasonography for gastric cancer N staging in this group were that the N0/N1 and overall diagnostic coincidence rates were high, reaching 88.89% and 81.81%, respectively, while the N2 diagnostic coincidence rates were low. It may be attributed to the study of Zhou and Li [27] that the detection rate of lymph nodes by ultrasound is related to the diameter of the lymph nodes. The larger the diameter, the higher the detection rate. Shimada et al. [28] also found that the detection rate of metastatic lymph nodes with a diameter of more than 0.5 cm is higher, but it is difficult to detect small lymph nodes with a diameter of less than 0.5 cm, especially less than 0.3 cm.

### 4.4. Evaluation of Gastric Filling Ultrasonography on M Stage of Gastric Cancer

Advanced gastric cancer is prone to metastasis. The common metastatic organs are the liver, lung, pancreas, peritoneum, and so on. Ultrasound has high-resolution for parenchymal organs, so it can accurately diagnose most metastatic organs. The coincidence rate of M0 and M1 in this group was high (100%), which was related to the location and size of the metastasis. However, small peritoneal metastases are easy to be missed, especially when there is no ascites.

### 4.5. Effect of Gastric Filling Ultrasonic Examination Stage on the Choice of Surgical Treatment

Nowadays, gastric cancer surgery is divided into reduced surgery (for the treatment of early gastric cancer), standard radical surgery and extended radical surgery (mainly for the treatment of advanced gastric cancer) and noncurative surgery (palliative treatment of advanced gastric cancer). D2 radical gastrectomy is regarded as the standard radical gastrectomy by most clinicians. According to the lymph node substation method of gastric cancer in Japan, no matter where the cancer focus is located in the stomach, the lymph nodes in groups No. 7, 8, and 9 are always the second station. Some people believe that the lymph nodes in groups No. 7, 8, 9, and 12 are also the stations most prone to skip metastasis [29, 30]. Therefore, we believe that we should first select the operation method according to the examination results before the operation. After the whole tumor and regional lymph nodes are removed, we should conduct a pathological examination for those with highly suspected metastasis of lymph nodes in groups No. 7, 8 and 9, which can help us determine the scope of lymph node dissection. If metastasis is confirmed, we will implement extended radical resection according to the general condition of the patient and whether there is distant metastasis. If no metastasis is confirmed, standard radical resection can be performed routinely. For extended radical operations (including D2 + 12 group lymph node dissection, D3 radical operation, and combined organ resection), most Japanese scholars believe that this operation can significantly improve the survival time of some patients with stage IIIB and IV [31], while European and American scholars represented by the Netherlands believe that this operation not only does not improve the survival time but also increases the incidence of complications [32]. Bonenkamp et al. [33] randomly investigated 1480 Dutch hospitals in terms of postoperative mortality and recurrence rate, and believed that extended radical mastectomy should not be widely used in western countries. The causes were analyzed and considered to be related to age, potential diseases such as cardiovascular and cerebrovascular diseases [34], obesity, doctors' surgical skills, and postoperative nursing [35].

## 5. Conclusion

In conclusion, the advantages of gastric filling ultrasonography in the diagnosis of gastric cancer lie in its high detection rate of lesions, high coincidence rate of T-stage of advanced gastric cancer, high detection rate of lymph nodes, and high coincidence rate of M-stage. The limitation is that its T-stage coincidence rate for early gastric cancer is low, and it is difficult to distinguish the relationship between tumor and surrounding inflammation, fibrosis, and scar tissue, which makes it easy to cause too deep judgment. In addition, it also has some limitations in the preoperative n-stage and the judgment of benign and malignant abdominal lymph nodes. However, because of its noninvasive, real-time dynamic, high-resolution, strong repeatability, and the good performance of gastrointestinal display AIDS, ultrasound can clearly show the lesions in the gastric cavity, gastric wall, and around the stomach, observe the depth of gastric wall infiltration, and accurately find the metastasis of extragastric lymph nodes and parenchymal organs. Gastric filling ultrasonography has high clinical practical value in the diagnosis of gastric cancer and its stages, and has a certain reference for the selection of surgical methods. However, the disadvantage of this study is that the sample size of the selected subjects is small, so we will expand the sample size for further research in the future and compare the diagnostic performance of gastric filling ultrasonography with other noninvasive diagnostic methods. It has been confirmed that gastric filling ultrasonography has application value in the evaluation of the condition of patients with gastric tumors and the selection of surgical treatment methods.

## Figures and Tables

**Figure 1:** ROC curve of T-stage of gastric cancer diagnosed by GFUS. *AZ* = 0.978, standard error = 0.016, and 95% confidence interval (0.946–1.00).

**Table 1:** Ultrasonic diagnosis and pathological results of gastric cancer (cases (%)).

Diagnostic method	Type	Gastric cancer	Nongastric cancer	Total
Ultrasonic	Gastric cancer	47 (94.00)	0	47 (94.00)
	Nongastric cancer	3 (6.00)	0	3 (6.00)

**Table 2:** Ultrasonic T-stage diagnosis results (cases (%)).

Pathological T-stage	Number of cases	Accuracy of ultrasonic diagnosis	Shallow judgment rate	Over depth judgment rate
T_1_	12	5 (41.67)	3 (25.00)	4 (T_2_ 33.33)
T_2_	7	4 (57.14)	0 (0.00)	3 (T_3_ 42.86)
T_3_	25	24 (96.00)	1 (T_2_ 4.00)	0 (0.00)
T_4_	6	5 (83.33)	1 (T_3_ 16.67)	0 (0.00)
Total	50	38 (76.00)	5 (10.00)	7 (14.00)

**Table 3:** Ultrasound assessment results of gastric mucosal thickness (‾median (range), mm).

Pathological T-stage	*n*	Full thickness median
T_1_-T_2_	19	9.80 (7.00–11.50)
T_3_-T_4_	31	17.00 (8.10–36.92)^#^

Note. Compared with T_1_-T_2_, ^#^*p* < 0.05.

**Table 4:** Ultrasonic *n*-stage diagnosis results (cases (%)).

Pathological N-stage	Number of cases	Coincidence rate of ultrasonic diagnosis	Noncoincidence rate of ultrasonic diagnosis
N_0_	18	16 (88.89)	2 (11.11)
N_1_	22	18 (81.81)	4 (18.18)
N_2_	10	7 (70.00)	3 (30.00)
Total	50	41 (82.00)	9 (18.00)

**Table 5:** Ultrasonic M-stage diagnosis results (cases (%)).

Pathological M-stage	Number of cases	Coincidence rate of ultrasonic diagnosis	Noncoincidence rate of ultrasonic diagnosis
M_0_	44	44 (100.00)	0 (0.00)
M_1_	6	6 (100.00)	0 (0.00)
Total	50	50 (100.00)	50 (100.00)

## Data Availability

The datasets during and/or analyzed during the current study are available from the corresponding author on reasonable request.
